This article has been retracted.

# Pancreatic cancer-initiating cell exosome message transfer into noncancer-initiating cells: the importance of CD44v6 in reprogramming

**DOI:** 10.1186/s13046-019-1129-8

**Published:** 2019-03-19

**Authors:** Zhe Wang, Hanxue Sun, Jan Provaznik, Thilo Hackert, Margot Zöller

**Affiliations:** 1 Department of Oncology, The First Affiliated Hospital of Guangdong Pharmaceutical University, Guangzhou, China; 2 Pancreas Section, University Hospital of Surgery, Im Neuenheimer Feld 110, D69120 Heidelberg, Germany; 3 Gene Core Unit, EMBL, Heidelberg, Germany

**Keywords:** CD44v6, Tspan8, Pancreatic cancer stem cells, Exosome biogenesis, Exosome message transfer, Non-cancer stem cell reprogramming

## Abstract

**Background:**

Cancer-initiating cell (CIC) exosomes (CIC-TEX) are suggested reprogramming Non-CIC. Mode of message transfer and engagement of CIC-markers being disputed, we elaborated the impact of CD44v6 and Tspan8 on the response of Non-CIC.

**Methods:**

Non-metastasizing CD44v6- and Tspan8-knockdown (kd) pancreatic cancer cells served as Non-CIC. CIC-TEX coculture-induced changes were evaluated by deep-sequencing and functional assays. Tumor progression was surveyed during in vivo CIC-TEX treatment.

**Results:**

Deep-sequencing of CIC-TEX-cocultured CD44v6kd-Non-CIC revealed pronounced mRNA changes in signaling, transport, transcription and translation; altered miRNA affected metabolism, signaling and transcription. CIC-TEX coculture-induced changes in Tspan8kd-Non-CIC mostly relied on CIC-TEX-Tspan8 being required for targeting. CIC-TEX transfer supported apoptosis resistance and significantly promoted epithelial mesenchymal transition, migration, invasion and (lymph)angiogenesis of the kd Non-CIC in vitro and in vivo, deep-sequencing allowing individual mRNA and miRNA assignment to altered functions. Importantly, CIC-TEX act as a hub, initiated by CD44v6-dependent RTK, GPCR and integrin activation and involving CD44v6-assisted transcription and RNA processing. Accordingly, a kinase inhibitor hampered CIC-TEX-fostered tumor progression, which was backed by an anti-Tspan8 blockade of CIC-TEX binding.

**Conclusions:**

This in depth report on the in vitro and in vivo impact of CIC-TEX on CD44v6kd and Tspan8kd Non-CIC unravels hub CIC-TEX activity, highlighting a prominent contribution of the CIC-markers CD44v6 to signaling cascade activation, transcription, translation and miRNA processing in Non-CIC and of Tspan8 to CIC-TEX targeting. Blocking CIC-TEX binding/uptake and uptake-initiated target cell activation significantly mitigated the deleterious CIC-TEX impact on CD44v6kd and Tspan8kd Non-CIC.

**Electronic supplementary material:**

The online version of this article (10.1186/s13046-019-1129-8) contains supplementary material, which is available to authorized users.

## Background

Pancreatic cancer (PaCa) has the highest cancer mortality rate and incidence is increasing [1]. High mortality, due to early spread and radio- and chemotherapy-resistance [2], is provoked by a small population of cancer-initiating cells (CIC) [3], which mainly act via exosomes (CIC-TEX) [4].

Exosomes (Exo), a subpopulation of small extracellular vesicles [5] are delivered by live cells [6]. They are composed of a lipid bilayer, integrated and membrane-attached proteins, some, prominently tetraspanins being engaged in Exo-biogenesis and -targeting [7]. The Exo plasma contains non-randomly recruited proteins, coating and non-coating RNA and DNA [6–9]. Exo components are function competent, message delivery severely affecting targets [10]. CIC-TEX reorganize the tumor stroma, stimulate angiogenesis, promote deviation of hematopoiesis towards immunosuppressive cells and transiently reprogram Non-CIC towards anchorage-independence, apoptosis-resistance, motility and invasion [11–14]. We focused on the CIC-TEX impact on Non-CIC, selecting cells with a knockdown (kd) of the PaCIC biomarkers CD44v6 (v6) and Tspan8 (Tsp8) as Non-CIC.

CD44v6 CIC-biomarker activity in PaCa [15] relies on the association with receptor tyrosine kinases (RTK), the engagement in Wnt signaling by associating with LPR6 (LDL receptor related protein 6)^1^ (see also Additional file 1: Table S1) and a contribution to NOTCH and Nanog epithelial-mesenchymal transition (EMT)-transcription factor activation [16–18]. CD44v6 also supports apoptosis-resistance, mostly via drug efflux, and facilitates tumor cell motility by protease transcription activation and protease proform cleavage promoting matrix remodeling [19, 20]. Regulation of miRNA processing adds to v6 CIC-biomarker activity [21, 22].

Metastasis-promoting Tsp8 [23] associations with integrins facilitates motile phenotype acquisition; protease links support path-creation for migrating tumor cells [24, 25]. The tetraspanin engagement in Exo-biogenesis and targeting is fundamental for the TEX-target crosstalk [26]. Tetraspanins connect with a multitude of transmembrane and cytosolic molecules in glycolipid-enriched membrane domains (TEM) [27]. TEM complexes, prone for internalization, are maintained during Exo biogenesis, TEX-Tsp8 most weightily forcing targeting [27–30].

Finally, there are two links between Tsp8 and v6. CD44v6 is Tsp8-associated in TEM and v6 promotes Tsp8 transcription [31, 32].

A v6kd and a Tsp8kd severely affecting PaCa progression [32–34], we aimed elaborating the molecular mechanism of v6 and Tsp8 in CIC-TEX activity. To achieve this goal, deep-sequencing (DS) was performed of CIC-TEX, untreated and CIC-TEX-treated v6kd and Tsp8kd cells. Correlating DS results with protein recovery and functional in vitro and in vivo studies uncovered v6 being central in CIC-TEX shaping. CIC-TEX, acting as hub initiating Non-CIC activation, profit from message delivery by Tsp8.

## Methods

### Tumor lines

The human PaCa lines A818.4 [35], Capan-1 [36], −v6kd and -Tsp8kd cells [32] and pcDNA3EGFP-Neomycin expression vector (Addgene) transfected A818.4 (A818.4-GFP < green fluorescence protein>) were maintained in RPMI1640/10%FCS/pyruvate/L-glutamine/antibiotics, transfected lines containing 0 .5mg/ml G418.

### Antibodies and reagents

Additional file 1: Table S2A, S2B.

### CIC-enrichment

Capan1-CIC were enriched by spheroid growth; A818.4-CIC by holoclone formation [32]. After 3 rounds of cloning, spheres/holoclones were cultured for 48 h in FCS-free medium. After 24 h recovery (medium with 10% Exo-depleted FCS), TEX were collected for an additional 48 h in FCS-free medium. Thereafter CIC-enriched cells were discarded.

### Tissue preparation

Nude mice were sacrificed by cervical dislocation or were anesthetized (CO_2_) collecting peripheral blood / peripheral blood leukocytes (PB, PBL) by heart puncture (100 U heparin/syringe). Tumors, liver, lung and hematopoietic / lymphoid tissues (bone marrow cells <BMC>, lymph node(s)/ <LN, LNC>, peritoneal exudate cells <PEC>, spleen cells <SpC>) were excised, shock frozen or dispersed.

### TEX preparation

Tumor cell supernatants were cleared (2x10min, 500 g, 1x20min, 2000 g, 1x30min, 10,000 g, 4 °C), filtered (0.22 μm) and centrifuged (120 min, 100,000 g, 4 °C). After washing (PBS, 120 min, 100,000 g, 4 °C), the pellet was resuspended in 40% sucrose overlaid by a discontinuous sucrose gradient (30–5%) and centrifuged (16 h, 100,000 g, 4 °C) collecting TEX from the 10–5% sucrose interface (light density fractions, d: 1.15–1. 56 g/ml) [28]. Protein concentrations were determined by Bradford. Where indicated, TEX were labeled with SP-DioC_18_(3) (3,3′-dioctadecyl-5,5′-di(4-sulfophenyl)oxacarbocyanine, Dio). After quenching (15 ml Exo-depleted FCS) and washing (2x120min, 100,000 g), TEX were suspended in 30 ml PBS layered over 10 ml 40% sucrose and centrifuged (120 min, 100,000 g, 4 °C), collecting the TEX-pellet at the bottom [28].

### mRNA and miRNA

Cell and TEX (RNase-pretreated) mRNA/miRNA were extracted using miRNeasyMinikit following the supplier’s suggestion (Qiagen, Hildesheim, Germany).

### mRNA and miRNA deep-sequencing

mRNA and miRNA DS of cells, TEX and TEX-treated cells were performed at the Core facility, EMBL, Heidelberg (ENA database accession No: PRJEB25446). Alignment software was STAR aligner version 2.5.2a, reference hg19. Differential recovery was defined by ≥1.5–2-fold changes in mean signal strength of normalized data.

### mRNA and miRNA analysis

PANTHER (http://pantherdb.org), KEGG (http://www.kegg.jp), Reactome (https://reactome.org), and STRING (http://string-db.org) databases were used for mRNA analysis. IPA (ingenuity program analysis) was used correlating miRNA with mRNA expression according to mRNA predictions (http://www.microrna.org, http://www.targetscan.org).

Real-time PCR (qRT-PCR) and delta-C_t_ method analysis followed described protocols [33] using GAPDH (mRNA) and small nuclear snRNA U6 (miRNA) as internal controls (primers: Additional file 1: Table S2C).

### Western blot (WB)

Lysates (cells: 30 μg, TEX: 10 μg) (30 min, 4 °C, HEPES buffer, 1% Lubrol or 1% TritonX-100, 1 mM PMSF, 1 mM NaVO_4_, 10 mM NaF, protease inhibitor mix) were centrifuged (13,000 g, 10 min, 4 °C), dissolved in Laemmli buffer and subjected to 10–12% SDS-PAGE. After protein transfer, blocking, blotting with antibodies, blots were developed with enhanced chemiluminescence (ECL) WB-detection-reagent. Relative signal strength in comparison to the actin control was evaluated by ImageJ. Where indicated significance between distinctly treated cell populations is indicated.

### Cell cycle analysis

Starved (48 h) and recovered (2 h, RPMI/10%FCS) cells were fixed (cold 70% ethanol, 1 h). After washing, propidium iodine (PI) (50 μg/ml, 3 .8mM Na citrate) was added (overnight, 4 °C), evaluating PI uptake by flow-cytometry.

### Apoptosis-resistance

The percent apoptotic cells (AnnV-APC/PI staining) after incubation (48 h) with cisplatin was determined by flow-cytometry.

### Flow-cytometry

TEX (10-15 μg) were coupled to 1 μl aldehyde-sulfate latex beads (LB) (4 μm) (Invitrogen) in PBS/1% BSA (90 min, 20 °C, shaking). After centrifugation, free binding site-blocking (100 mM glycine in PBS, 1 h) and two washings (PBS/1%BSA), TEX-coated beads were distributed in 96-well plates. Staining with primary and secondary dye-labeled antibodies followed the protocol for cell staining. For intracellular staining, cells/TEX were fixed and permeabilized. Samples were analyzed in a FACSCalibur using the CellQuest program.

### Immunohistochemistry

Shock-frozen tissue sections (8 μm) were fixed, incubated with antibodies, washed, exposed to biotinylated secondary antibodies and alkaline phosphatase-conjugated avidin-biotin solution. Sections were counter-stained with hematoxilin. Digitized images were generated using a Leica DMRBE microscope.

### Confocal microscopy

Cells were seeded on cover-slides, tissue sections on glass-slides. Cells/tissues were fixed, permeabilized, blocked, incubated with primary antibody, washed, incubated with fluorochrome-conjugated secondary antibody and counterstained with DAPI. Slides were mounted in Elvanol. Digitized images were generated using a Leica LMS800 microscope and Carl Zeiss Vision software for evaluation.

### Animal experiments

Nude mice received orthotopic (ot) or subcutaneous (sc) tumor cell injections. When tumors (sc) reached a mean diameter of 0 .5cm or became palpable (upper abdomen), tumor-bearing (TB) and control mice received an intravenous (iv) injection of 100 μg SP-DioC_18_(3) labeled TEX or GFP-transfected cell-derived TEX (TEX-GFP), sacrificing 3 mice/group after 2 h–48 h. Where indicated, mice received tumor injections on the left and right upper back or received iv injections of TEX (200 μg/100 μl NaCl, 1x or 2x/wk), or anti-Tsp8 (200 μg/100 μl NaCl, weekly) or Gemcitabine (GEM) (100 μg/g, weekly). Mice (5–6/group) were sacrificed tumors reaching 1 .5cm mean diameter or upon weight loss. Animal experiments were Government-approved (Baden-Wuerttemberg, Germany).

### Statistics

In vitro experiments were repeated 3-times; in vivo experiments 2-times. *P* values < 0.05 (two-tailed Student’s t-test, Kruskal-Wallis test, where indicated after Bonferroni-Holm correction) were considered significant and are indicated by * or s or *p*-values are presented.

## Results

CIC-TEX transfer CIC features into Non-CIC, the contribution of CIC-biomarkers and the consequences of transfer being disputed. We approached the question using A818.4 CIC-TEX and A818.4-v6kd and -Tsp8kd cells as Non-CIC, both kd strongly impairing tumor progression [25, 32]. In vitro assays, based on DS analyses, were substantiated by in vivo studies of CIC-TEX-treated TB mice.

### CIC-TEX binding/uptake and metastatic growth induction in CD44v6kd and Tspan8kd cells

Binding and uptake of CIC-TEX is a prerequisite for Non-CIC modulation. A818.4 cells and TEX abundantly express v6 and Tsp8 with a mutual effect of a v6kd and, less pronounced, a Tsp8kd. A v6kd also affects MET and a Tsp8kd CD104 expression (32). Flow-cytometry analysis validated v6 and upregulated Tsp8 recovery in TEX. Characterization for common TEX markers confirmed high expression of Alix, TSG101, MFG8 and tetraspanins with only a minor reduction of CD63 in v6kd TEX (Additional file 1: Figure S1a). To control for TEX uptake in vivo, intrapancreatic TB mice received an iv Dio-labeled TEX injection. A818.4, −v6kd and -Tsp8kd cells take-up TEX with comparable efficacy, uptake increasing until 24 h after injection. In the tumor-free pancreas, TEX are transiently recovered at low level. TEX are also recovered in draining LN, BM, lung, liver, spleen and PB (Additional file 1: Figure S1b, S1c). The experiment was repeated with weekly iv GFP-TEX injections into sc A818.4 and -v6kd TB. Tumors and metastasis-prone organs were excised, tumors reaching 0 .5cm mean diameter. GFP was mostly recovered in Tsp8+ dispersed tumor tissue and draining LN (Additional file 1: Figure S1d). Confocal microscopy of shock-frozen tumor sections confirmed GFP-TEX uptake by Tsp8+, VEGFR2+ and VEGFR3+ v6kd tumor cells, TEX particularly colocalizing with Tsp8. TEX were also taken-up by mouse endothelial cells (EC) (Additional file 1: Figure S1e). GFP+ non-tumor cells in BM and lung were mostly and in the liver exclusively CD11b + mouse monocyte (Mϕ) (Additional file 1: Figure S1f). Thus, CIC-TEX uptake is unimpaired in v6kd and Tsp8kd Non-CIC.

The impact of CIC on distant Non-CIC was evaluated injecting A818.4-GFP-CIC in the upper left and A818.4-v6kd cells in the upper right back. A818.4-GFP-CIC promoted A818.4-v6kd cell growth, differences being first seen 4wk after tumor cell application (Fig. 1a). Flow-cytometry revealed very weak green fluorescence in dispersed v6kd tumor cells that were Tsp8+, EpC+ and faintly v6+ (Fig. 1b,c). Iv injected CIC-TEX also promoted A818.4-v6kd and -Tsp8kd cell intrapancreatic growth resulting in a significant survival time reduction (Fig. 1d), a strong increase in tumor cell dissemination (peritoneal cavity, PB) and in LN, spleen, BM, liver and lung settlement, evaluated by tumor cell outgrowth during ex vivo culture, the cumulated number of organs with disseminated tumor cells differing significantly (Fig. 1e).

**Fig. 1:** The impact of CIC-TEX on CD44v6kd and Tspan8kd tumor growth and progression. **a**-**c** Nude mice received GFP-transfected A818.4 CIC on the left upper back and/or A818.4-v6kd cells on the right upper back. **a** Mean tumor diameter ± SD (3mice/group); **b**,**c** mean percent GFP+, GFP + marker+ and marker+ (v6, Tsp8, EpC) cells was evaluated at autopsy (flow-cytometry); **a**-**c** significant differences between mice receiving only CD44v6kd cells and mice receiving a contralateral injection of CIC-GFP: s. **d**,**e** Nude mice received an ot injection of 1 × 10^6^ wt or v6kd or Tsp8kd cells and weekly 200 μg/mouse CIC-TEX, iv; **d** survival time and mean survival time of 6 and 5, respectively, mice/group; *p*-values comparing wt versus kd tumor and kd tumor depending on CIC-TEX application are indicated. **e** The indicated organs, collected at autopsy, were dispersed and maintained in culture to observe tumor cell outgrowth; p-values (Kruskal-Wallis after Bonferroni-Holm correction) for the total No of organs with disseminated tumor cells are indicated comparing wt versus kd TB mice and CIC-TEX-treated kd TB mice. After reaching a mean tumor diameter of ~ 0 .5cm, CIC assist the growth of v6kd Non-CIC, likely via delivery of TEX. The shortened survival time and the increase in disseminated tumor cells of v6kd TB mice receiving CIC-TEX supports this assumption

CIC-TEX sufficing to partially rescue metastatic capacity of v6kd and Tsp8kd cells, we searched for the molecular mechanism(s) underlying CIC-TEX activity.

### CIC-TEX affect the CD44v6kd and Tspan8kd non-CIC mRNA and miRNA profile

The impact of CIC-TEX on kd cells was evaluated by DS of mRNA and miRNA after 72 h coculture.

A818.4, −v6kd and -Tsp8kd cells contained between 1381 to 1578 mRNA with a signal strength ≥5000. Panther pathway molecular function analysis revealed a slightly increased number of structural molecules in the kd cells (Additional file 1: Figure S2a). A818.4-wt cells and TEX also displayed similar molecular function patterns (Additional file 1: Figure S2b). Nonetheless, CIC-TEX significantly affected individual gene expression in v6kd cells (278 upregulated; 255 downregulated mRNA) and, less pronounced, Tsp8kd cells (51 upregulated; 63 downregulated mRNA) (≥1000 signal strength, ≥2.0 fold-change) (Additional file 1: Table S3A-S3D and Figure S2c). Sorting distinctly recovered mRNA in CIC-TEX-treated v6kd cells according to transcription/translation, transport, oncogenesis, angiogenesis, apoptosis, adhesion/proteolysis and signaling with a focus on EMT (Reactome database) showed a dominance of up- or downregulated signaling-engaged mRNA, followed by RNA engaged in transport and transcription/translation including splicing. In CIC-TEX-treated Tsp8kd cells changes in signaling-engaged mRNA also holds the leading position (Additional file 1: Figure S2d, S2e).

The molecular mechanism of TEX activity being debated, we controlled for a direct mRNA transfer from CIC-TEX into targets. Only 19 of 51 upregulated mRNA in Tsp8kd and 60 of 278 upregulated mRNA in v6kd cells were ≥ 2.0-fold higher in CIC-TEX than untreated kd cells (Fig. 2a). Similarly, a considerable number of mRNA ≥2.0-fold downregulated after coculture with CIC-TEX (Tsp8kd: 63 mRNA, v6kd: 255 RNA in cells) were recovered at an ≥2.0-fold higher level in CIC-TEX than kd cells, the random correlation between CIC-TEX and CIC-TEX-treated kd cell mRNA being shown for v6kd cells (TEX and/or v6kd cell signal strength ≥1000) (Additional file 1: Table S3E). Additional file 1: Table S3F presents mRNA of CIC-TEX-treated Tsp8kd cells that expression was upregulated by CIC-TEX treatment (signal strength of at least one component ≥1000, fold-change in untreated versus CIC-TEX-treated Tsp8kd cells: ≥2.0); mRNA recovery in CIC-TEX is included and ≥ 2.0-fold higher mRNA recovery in both CIC-TEX and CIC-TEX-treated Tsp8kd cells is indicated in bold (Additional file 1: Table S3F). The rare correlation between recovery in CIC-TEX and CIC-TEX-treated kd cells argues against transferred mRNA directly accounting for changed CIC-TEX-treated kd cell mRNA profiles.

**Fig. 2:** Correlation between CIC-TEX and CIC-TEX-induced changes in mRNA and miRNA profiles. **a** Numbers of ≥2-fold enriched mRNA (signal strength ≥1000) in CIC-TEX-treated v6kd and Tsp8kd cells sorted according to ≥2-fold higher versus comparable or lower recovery in CIC-TEX than kd cells; **b** numbers of miRNA ≥1.5-fold upregulated in CIC-TEX-treated v6kd and Tsp8kd cells sorted according to ≥1.5-fold higher versus comparable or lower recovery in CIC-TEX than kd cells; **c** Correlation between ≥1.5-fold up- or downregulated mRNA in CIC-TEX treated v6kd and Tsp8kd cells sorted according to reverse miRNA recovery in CIC-TEX-treated cells; **d** major activities (IPA-based Reactome analysis) of ≥2-fold up- or downregulated mRNA that are predicted targets of inversely recovered miRNA (miRNA database, target scan database) in both CIC-TEX-treated v6kd and Tsp8kd cell (List of synonyms: Additional file 1: Table S1). mRNA and miRNA recovery are more strongly affected by CIC-TEX treatment in CD44v6kd than Tsp8kd cells. However, at the mRNA and the miRNA level coculture-induced changes rarely correlate with the CIC-TEX content. Instead, there is a strong correlation between coculture-induced up- or downregulated miRNA and reversely down- or upregulated mRNA in CIC-TEX-treated kd cells, indicating that not the CIC-TEX content, but CIC-TEX-induced target cell activation is dominating

Alternatively, transferred miRNA could account for mRNA downregulation. The impact of a v6kd or a Tsp8kd in cells and TEX on miRNA recovery were described (Sun H. et al., submitted). These studies, performed with miRNA arrays, cannot be directly compared to the DS analyses. With the current focus on the impact of CIC-TEX, we just want to mention that a v6kd more strongly affects miRNA recovery in cells and TEX than a Tspa8kd, which is shown for miRNA with a signal strength of > 1000 in TEX, where a reduction in let7-miRNA in v6kd-TEX is dominating (Additional file 1: Figure S3a, S3b). The comparison of miRNA in CIC-TEX versus v6kd or Tsp8kd cells revealed 97 miRNA (signal strength ≥500) showing ≥1.5-fold higher signal strength in CIC-TEX than the kd cells and an ≥1.5-fold increase in signal strength of 46 miRNA in kd cells after CIC-TEX treatment (Additional file 1: Table S4A, S4B and Figure S3c,S3e). Despite qRT-PCR providing evidence for miRNA transfer from CIC-TEX into target cells (Additional file 1: Figure S3d), an ≥1.5-fold increase in CIC-TEX-treated kd cells rarely correlated with an ≥1.5 higher recovery in CIC-TEX than kd cells (Fig. 2b). Changed miRNA recovery poorly reflecting transferred CIC-TEX miRNA was supported by 30 miRNA downregulation in CIC-TEX-treated v6kd and/or Tsp8kd cells (Additional file 1: Table S4C and Figure S3f). However, within CIC-TEX-treated kd cells co-culture-induced increased and reduced miRNA correlated in ≥50% with changed mRNA expression of predicted targets (http://www.microrna.org, http://www.targetscan.org) (Additional file 1: Table S5A, S5B, Fig. 2c). Reactome analysis of predicted mRNA targets of a coculture-promoted ≥2-fold increase or decrease in both v6kd and Tsp8kd cells and an inverse regulation of miRNA in v6kd and/or Tsp8kd cells pointed towards transcriptional regulation-engaged mRNA being released from repression; signaling-engaged mRNA being up- or downregulated and metabolism-engaged mRNA frequently being targets of upregulated miRNA (Fig. 2d).

These findings are hardly compatible with transferred CIC-TEX mRNA or miRNA directly accounting for Non-CIC reprogramming, but support CIC-TEX providing a hub in core signal transducer activation and/or a shift in the metabolic state. Being concerned about the crosstalk between CIC-TEX and v6kd or Tsp8kd Non-CIC, the hypothesis was only surveyed for pronounced changes in signal transduction and selected features of tumor progression impaired in v6kd and/or Tsp8kd Non-CIC.

### CIC-TEX-promoted signaling, apoptosis-resistance, EMT, motility and invasion in non-CIC

A signaling array revealed CIC-TEX-promoted activation of EGFR, Erb2, Erb3, InsR, IGF1R, TrkA1 and -A2, Ron, RET, EphA1, EphB3, Tyro3, Tie2 and VEGFR2 in v6kd cells. The impact of CIC-TEX on A818.4-Tsp8kd cells was partly overlapping. TRKA1, −A2, Tyro3 and TEK did not, FGFR1, − 3, − 4 and MCSFR became only upregulated in Tsp8kd cells (Fig. 3a, Additional file 1: Figure S4a and Table S1). Flow-cytometry and WB confirmed upregulated EGFR, HER2, EphA1, VEGFR1/2/3 and PDGFRB expression, where representative examples are presented for the WB and relative signal strength compared to the actin control of 3 independently performed experiments as well as the *p*-values of kd cells versus CIC-TEX-treated kd cells are included (Fig. 3b,c, Additional file 1: Figure S4b and Table S1). Flow-cytometry analysis indicated src, FAK, ras, rac, jun and IκB activation by CIC-TEX, although in some instances v6kd- and Tsp8kd-TEX also exerted weak effects. WB analysis, representative examples and statistical evaluation of 3 independently performed WB confirmed the flow-cytometry results (Fig. 3d,e, Additional file 1: Figure S4c and Table S1).

**Fig. 3:** CIC-TEX-initiated changes in RTK and downstream signaling molecules in CD44v6kd and Tspan8kd cells. **a** Signaling array of A818.4-v6kd cells cultured for 72 h with/without CIC-TEX. The relative signal strength was evaluated by ImageJ; significant differences by coculture with CIC-TEX: *. Flow-cytometry and WB analysis of (**b**,**c**) RTK expression in kd-TEX- or CIC-TEX-treated kd cells and (**d**,**e**) major pathway-engaged cytosolic signaling molecules; **b**,**d** mean % stained cells±SD (3 assays), significant differences by coculture with TEX: *; **c**,**e** representative examples and relative signal strength±SD of 3 independent experiments including p-values for kd cells compared to CIC-TEX-treated kd cells; **f** pathways from miRNA to RTK (IPA-based STRING analysis after predicted target mRNA selection by microrna.org and targetscan.org) for ≥2-fold upregulated miRNA (framed) and ≥ 2-fold reduced mRNA recovery in CIC-TEX-treated v6kd or Tsp8kd cells compared to untreated kd cells; **g** IPA-based STRING analysis after predicted target mRNA selection by microrna.org and targetscan.org for ≥2-fold reduced miRNA in CIC-TEX-treated compared to untreated v6kd cells and of ≥2-fold upregulated predicted mRNA targets that are engaged in signal transduction. **h** Flow-cytometry analysis of ex vivo harvested intrapancreatic A818.4-v6kd cells from nude mice with/without weekly iv CIC-TEX treatment; mean % stained cells±SD (3 tumors), significant differences by CIC-TEX treatment: s; **i** Representative immunohistology examples of A818.4-v6kd and -Tsp8kd shock-frozen tumor sections with/without CIC-TEX treatment stained with the indicated antibodies (scale bar: 100 μm). (List of synonyms: Additional file 1: Table S1). CIC-TEX treatment strongly affects RTK expression and downstream signaling molecules in vitro and in vivo. Changes in the recovery of mRNA engaged in signal transduction (Additional file 1: Figure S2d, S2e) are accompanied at a noteworthy frequency by reversely altered miRNA expression in CIC-TEX-treated kd, predominantly v6kd cells

Several miRNA ≥2-fold upregulated in CIC-TEX-treated v6kd and/or Tsp8kd cells target mRNA that are engaged in RTK signaling and mRNA expression was reduced after coculture (Additional file 1: Table S5A). After coordinating miRNA that was upregulated in v6kd or Tsp8kd cells after CIC-TEX treatment with predicted target mRNA that became ≥2-fold downregulated and searching selectively for an engagement in RTK pathways by IPA-based STRING analysis revealed in CIC-TEX-treated v6kd and Tsp8kd cells Spry (sprouty RTK signaling antagonists) 4, interfering with multiple signal transduction molecule activation [37], as the central target for upregulated miRNA in both CIC-TEX-treated kd lines (Fig. 3f). More striking was the correlation between ≥2-fold reduced miRNA and ≥ 2-fold increased predicted mRNA target recovery in the CIC-TEX-treated kd cells (Additional file 1: Table S5B). In v6kd and Tsp8kd cells 8 miRNA with ≥2-fold reduced expression after coculture have four predicted signaling molecule target mRNA, which became ≥2-fold upregulated after coculture. Only DCBLD2 (discoidin, CUB and LCCL domain containing 2) and NRP1 (neuropilin1) are predicted targets of three miRNA. DCBLD2 is a scaffold receptor expression being associated with invasiveness [38]. Expression of the CIC marker NRP1 accounts for higher clonogenicity, self renewal potential and migratory activity [39]. An additional five miRNA, displaying ≥2-fold reduced expression in CIC-TEX-treated Tsp8kd cells had 8 predicted signaling engaged target mRNA that expression level became ≥2-fold increased, the upregulated mRNA being predicted targets of only one or two downregulated miRNA (Additional file 1: Figure S4d). Instead, in CIC-TEX-treated v6kd cells additional 29 signal transduction-engaged mRNA with ≥2-fold upregulated expression were predicted targets of 24 miRNA recovered at an ≥2-fold decreased level. Many of these repression released mRNA were targets of several miRNA recovered at an ≥2-fold lower level in CIC-TEX-treated than untreated v6kd cells. The most prominent likely repression-released target was CDK6 (cyclin-dependent kinase 6), which is not shown as it predominantly regulates G1 phase progression and G1/S transition, altered expression being frequently observed in cancer [40] (Fig. 3g).

In vivo CIC-TEX treatment sufficed for EGFR, PDGFRB, EphA4, VEGFR2 and NGFR upregulation in A818.4-v6kd cells and, distinct to the coculture, MAPK pathway activation (Fig. 3h). Immunohistology confirmed pronounced VEGFR2/3, PDGFRB, EGFR and EphA4 expression in v6kd and Tsp8kd tumors of CIC-TEX-treated mice, PDGFRB becoming particularly upregulated in v6kd tumors (Fig. 3i). More pronounced activation in tumor tissue than in cocultures could be a sequel of persisting stimulation and a feedback by the tumor stroma.

Confirming DS analyses, protein and functional in vitro and in vivo studies suggest RTK and signaling cascade activation relying, at least partly, on CIC-TEX binding-initiated activation. Upregulation of miRNA that repress signaling-inhibiting mRNA and miRNA downregulation allowing for mRNA release from repression provide an independent supplemental input, the dominance of v6 probably resting on its engagement in mRNA and miRNA processing [33]. The strong impact of CIC-TEX on v6kd cells in modulating miRNA engaged in RTK and downstream signaling pathways activation demands putting emphasis on unequivocally answering the mode of action.

Apoptosis-resistance being a central CIC feature, we proceeded searching for the impact of transferred CIC-TEX on apoptosis resistance of v6kd and Tsp8kd cells cultured for 48 h in the presence of cisplatin. Reduced apoptosis resistance of v6kd and Tsp8kd cells being partially corrected by CIC-TEX coculture (Fig. 4a), hints towards the underlying molecular processes were searched for by DS, controlling for selected proteins in vitro and ex vivo by flow-cytometry and immunohistochemistry.

**Fig. 4:** CIC-TEX-promoted apoptosis-resistance in CD44v6kd and/or Tspan8kd cells. **a** Flow-cytometry of cells cultured for 48 h in the presence of cisplatin; mean % AnnexinV+ and AnnexinV+/PI+ cells±SD (triplicates); significant differences of wt cells versus CIC or kd cells: *; significant differences by CIC-TEX treatment: s. **b** mRNA that expression differed by ≥2-fold after CIC-TEX treatment in Tsp8kd (blue) or v6kd (violet) cells were sorted by KEGG analysis according to the engagement in distinct apoptotic processes. **c**-**f** Flow-cytometry analysis of apoptosis-related receptor and cytoplasmic signaling molecules in A818.4, −v6kd and CIC-enriched cells and in v6kd cells cocultured with v6kd- or CIC-TEX; mean % stained cells±SD (3 assays), significant differences between wt cells, v6kd cells and CIC: *, significant differences by coculture of v6kd cells with TEX: s. **g** Representative immunohistology examples of A818.4 and -v6kd shock-frozen tumor sections from untreated or CIC-TEX-treated mice stained with the indicated antibodies (scale bar: 100 μm). (List of synonyms: Additional file 1: Table S1). Slightly reduced apoptosis resistance of v6kd and Tsp8kd tumor cells becomes mitigated by CIC-TEX treatment. The impact of CIC-TEX on apoptosis resistance is mostly restricted to the regulation of molecules engaged in the intrinsic pathway of apoptosis induction. An exception is the increased expression of drug transporters in CIC-TEX-treated v6kd cells

Sorting by Reactome analysis in v6kd and Tspan8kd cells for apoptosis-related mRNA that expression was ≥2-fold altered after coculture with CIC-TEX according to the engagement in regulation of apoptosis, receptor-mediated or intrinsic apoptosis pathways revealed a predominant contribution of mRNA engaged in apoptosis regulation. Notably, Hyal2 (hyaluronoglucosaminidase 2) [41, 42] became down- and Dicer [43] upregulated in CIC-TEX-treated v6kd cells. Hardly any contribution of mRNA engaged in receptor-mediated apoptosis was seen and only few mRNA involved in the intrinsic apoptosis pathway were affected. Most notably was the upregulation of ABC (ATP binding cassette) drug transporters that was only observed in v6kd cell cocultures with CIC-TEX (Fig. 4b). Predicted targets of miRNA engaged in apoptosis/apoptosis regulation were searched by the microrna.org and targetscan.org program. Though ≥2-fold up- or downregulated miRNA and mRNA frequently inversely correlated, only few predicted mRNA were targets of at least 3 miRNA. These included the downregulated mRNA CDKN1A/p21 (cyclin dependent kinase inhibitor 1A) [44], CLU (clusterin) [45], DHCR24 (24-dehydrocholesterol reductase) [46], SFN (stratifin) [47], STAT1 [48], TGM2 (transglutaminase 2) [49] and VEGFB [50], mostly engaged in apoptosis regulation and rarely in intrinsic apoptotic signaling. NGFR (nerve growth factor receptor) also is engaged in death receptor signaling [51]. Only upregulated EMP1 (epithelial membrane protein 1) and PMAIP1 (phorbol-12-myristate-13-acetate-induced protein 1), engaged in regulation of the intrinsic apoptosis pathway and apoptosis execution [52, 53], are predicted targets of several downregulated miRNA. Thus, none of the potential miRNA targets plays a central role in apoptosis. Notably, drug transporter mRNA was not a predicted target of any miRNA showing altered expression in CIC-TEX-treated v6kd and Tsp8kd cells (Additional file 1: Figure S5a, S5b).

A Tsp8kd having a minor impact, CIC-TEX correction of apoptosis-resistance at the protein level is only shown for v6kd cells exhibiting slightly upregulated actCasp3 and cleaved Casp9 and reduced MDR1, pAkt and pBAD expression (Fig. 4c,d). CIC-TEX treatment uncovered pAkt, Bcl2, BclXl upregulation and a minor BAX reduction, dominating being MDR1 upregulation (Fig. 4e,f). The impact of CIC-TEX on apoptosis-related genes became stronger in vivo. Immunohistochemistry of v6kd tumor sections revealed upregulated Casp3 and Casp9 being reduced and reduced TNFRI, AIF and MDR1 expression being rescued in CIC-TEX-treated v6kd-TB mice (Fig. 4g).

CIC-TEX hardly affected receptor-mediated apoptosis and apoptosis-executing molecules, but rescued ABC transporter expression in v6kd cells. A minor contribution of CIC-TEX to PI3K/Akt pathway activation likely accounts for v6kd and Tsp8kd cells. CIC-TEX-promoted changes in miRNA have a mean impact on apoptosis-resistance, predicted mRNA frequently are potential targets of only one or two miRNA. The stronger effects of CIC-TEX treatment in vivo point towards additive support by the tumor surrounding. Nonetheless, the less impressive changes by CIC-TEX treatment of v6kd and Tsp8kd cells fit to the weak impact of CIC-TEX on apoptosis resistance.

CIC-TEX can promote EMT, which beside others supports anchorage-independent growth, evaluated by colony formation in soft agar. Anchorage-independent growth of v6kd and Tsp8kd cell was strongly reduced compared to wt cells, but was rescued in cultures containing CIC-TEX, but not v6kd- or Tsp8kd-TEX (Fig. 5a). CIC also are characterized by slow cell cycle progression, which was evaluated after synchronization (48 h starving) by PI uptake. Cell cycle progression was accelerated in v6kd and Tsp8kd cells compared to CIC and became significantly retarded in CIC-TEX-treated kd cells (Fig. 5b).

**Fig. 5:** The impact of CIC-TEX on EMT gene expression. **a** Tumor cells were seeded in soft agar containing 30 μg/ml TEX, where indicated; mean No of colonies±SD (5 replicates) and representative examples after 3wk of culture; **b** cell cycle progression (flow-cytometry, PI staining) of wt, CIC and kd cells cultured with/without CIC-TEX; mean % of cells (5 replicates) in G0, G1/S and G2/M; **c** IPA-based Reactome analysis of transcription factor-, stem cell-, EMT-, transcription-, and EMT-regulating genes that mRNA level is ≥2-fold up- or downregulated in CIC-TEX-treated v6kd and Tsp8kd cells (red), Tsp8kd cells (blue) or CD44v6kd cells (violet). **d**,**e** Reactome analysis after IPA coordination of miRNA with predicted mRNA targets (miRNA and targetscan databases) of (**d**) > 2-fold upregulated miRNA (framed) and (**e**) downregulated miRNA in CIC-TEX-treated kd cells affecting EMT-related genes in kd cells; in (**d**) mRNA pathways from upregulated miRNA towards EMT are included; for downregulated miRNA (**e**) only direct predicted mRNA targets are shown (color code as in c). **f** Flow-cytometry of EMT markers in A818.4 and kd cells with/without CIC-TEX-treatment (72 h); **g** confocal microscopy of kd cells with/without CIC-TEX-treatment stained for E- or N-cadherin and counterstained for v6 or Tsp8 (scale bar: 10 μm); **h** Flow-cytometry of ex vivo analyzed EMT markers in dispersed intrapancreatic v6kd tumors from mice with/without CIC-TEX-treatment; (**i**) Flow-cytometry of EMT-related transcription factors in A818.4 and kd cells with/without CIC-TEX-treatment (72 h); **j** Confocal microscopy of kd cells with/without CIC-TEX-treatment stained for EMT-related transcription factors NOTCH and Nanog and counterstained with anti-v6 or anti-Tsp8 (scale bar: 10 μm); **f**,**h**,**i** mean % stained cells±SD (3 assays/tumors); **a**,**b**,**f**,**h**,**i** significant differences between wt and kd cells: *, significant differences by CIC-TEX-treatment: s. (List of synonyms: Additional file 1: Table S1). CIC-TEX partly rescue impaired anchorage-independent growth and accelerate kd cell cycle progression. DS, confirmed at the protein level, unraveled a strong impact of CIC-TEX on EMT-related transcription factors mostly in v6kd cells at the mRNA and miRNA level, the latter being particularly engaged in Wnt and NOTCH signaling

DS analysis of EMT marker and EMT-related transcription factor expression indicated low signal strength (< 500) for most EMT markers and EMT-regulating transcription factors. Nonetheless, NOTCH1, TWIST1, LPR6 and SOX4 were ≥ 1.5-fold upregulated in CIC-TEX-treated v6kd cells (data not shown). However, IPA-based Reactome analysis uncovered a significant number of transcription factors and transcription regulating mRNA as well as of mRNA engaged in Wnt and, less frequently NOTCH, BMP and SCF-Kit signaling that expression was ≥2-fold changed, predominantly in v6kd cells after CIC-TEX coculture. Notably, expression of 6 mRNA, explicitly engaged in EMT regulation, was reduced in CIC-TEX-treated v6kd cells. Expression of only few mRNA was ≥2-fold up- or downregulated in both v6kd and Tsp8kd cells or in Tsp8kd cells after CIC-TEX treatment. EMT-related activities of these latter mRNA corresponded to those described for CIC-TEX-treated v6kd cells (Fig. 5c).

There is additional evidence for a possible contribution of miRNA to EMT regulation. Eight, respectively, seven miRNA with ≥2-fold increased recovery in CIC-TEX-treated v6kd and Tsp8kd cells concomitantly displayed ≥2-fold downregulation of EMT-related predicted target mRNA. The bHLH MYCL (MYC lung carcinoma derived homolog) transcription factor [54] appears to be central in modulating EMT in v6kd cells in response to CIC-TEX-promoted miRNA upregulation. In Tspan8kd cells the transglutaminase TGM2, promoting apoptosis resistance and tumor progression [55], is a predicted target by several CIC-TEX-promoted upregulated miRNA (Fig. 5d). On the other hand, a higher number of miRNA that have predicted mRNA targets engaged in the EMT process were expressed at an ≥2-fold reduced level after CIC-TEX coculture, where CDK6, CSNK1A1 (casein kinase 1 alpha 1) and PPP3CA (protein phosphatase 3 catalytic subunit alpha) are predicted targets of several miRNA. CDK6 is primarily engaged in cell cycle regulation [56], the impact on EMT remaining to be further explored. However, STRING analysis revealed that 10 of 15 mRNA possibly released from miRNA repression in the v6kd and/or Tsp8kd cells, including CSNK1A1 [57] and PPP3CA [58] are engaged in Wnt and 4 in NOTCH signaling (Fig. 5e).

Protein analysis confirmed unaltered E-cadherin and vimentin expression in the v6kd and Tsp8kd Non-CIC irrespective of CIC-TEX coculture. CIC-TEX rescued reduced N-cadherin expression in v6kd and Tsp8kd cells and reduced fibronectin (FN) expression in Tsp8kd cells (Fig. 5f). Confocal microscopy endorsed unaltered E-cadherin expression in the CIC-TEX-treated kd cells and pronounced colocalization with v6; CIC-TEX-promoted upregulated N-cadherin also preferentially colocalized with v6 (Fig. 5g). Upregulated N-cadherin, but unaltered E-cadherin, FN and vimentin expression was also seen in ex vivo analyzed dispersed v6kd tumor tissue from CIC-TEX-treated mice (Fig. 5h). Protein analysis confirmed CIC-TEX coculture mostly rescuing reduced NOTCH and Nanog expression in v6kd and Tsp8kd cells and Slug, Snail, Twist and Wnt5a/b expression in v6kd cells (Fig. 5i), confocal microscopy affirming for NOTCH and Nanog colocalization with v6 and Tsp8 (Fig. 5j).

CD44v6 and Tspan8 contribute to tumor cell motility and invasion and defects of v6kd and Tspan8kd cells are corrected by CIC-TEX. The contribution of Tspan8 relies on its association with integrins, driving beside others α6β4 out of hemidesmosomes into TEM, where integrins become activated promoting cytosolic signaling molecule activation that allows for lamellipodia and focal adhesion point generation. Tspan8 also is engaged in protease activation mostly via associated membrane-anchored MMP [25, 34]. CD44v6 promotes activation of protease transcription and protease proform cleavage, which facilitates generating space for migrating tumor cells [32, 59]. These findings being already demonstrated for A818.4-v6kd and -Tspan8kd cells as well as the partial correction of deficits by CIC-TEX [32, 34], the question on the correlation with the DS analysis remained to be answered.

We evaluated at the mRNA level proteases and adhesion molecules that were upregulated after coculture of v6kd or Tspan8kd cells with CIC-TEX by ≥1.5-fold. Excluding the proteasome, comparably few proteases were distinctly recovered with a surprisingly high percentage of protease inhibitors. This accounted for CIC-TEX-treated v6kd and Tsp8kd cells. Adhesion molecule analysis, restricted to membrane-anchored and cytoskeleton interacting proteins (ligands indicated in brackets) revealed CIC-TEX treatment fostering integrin, laminin, cadherin- and actin-interacting protein expression (Fig. 6a). STRING pathway analysis of adhesion molecule RNA with upregulated expression after CIC-TEX treatment uncovered predominant upregulation of integrin-, GPCR- and RTK-signaling pathway components, indicated in brackets, in v6kd cells (Fig. 6b).

**Fig. 6:** CIC-TEX engagment in protease, adhesion molecule and related signaling regulation in CD44v6kd and Tspan8kd cells. **a** CIC-TEX coculture-induced ≥1.5-fold upregulated RNA expression was analyzed by KEGG for engagement in proteolysis and adhesion. The analysis was restricted to plasma membrane or plasma membrane attached proteins; proteases and inhibitors (indicated in brackets) are listed for migration; for adhesion molecules the predominant ligands are included in brackets. **b** Assignment of major adhesion / motility promoting signaling molecules (STRING analysis) that expression was ≥1.5-fold upregulated by CIC-TEX coculture; major targets are indicated in brackets. (Abbreviations: AJ: adherens junction, cadh: cadherin, chemok: chemokine, coll: collagen, CS: chondroitin sulphate, cytosk: cytoskeleton, FN: fibronectin, GPCR: G-protein coupled receptor, growthF: growth factors, HA: hyaluronan, inhib: inhibitor, int: integrin, LN: laminin, Synd: syndecan, List of synonyms: Additional file 1: Table S1). CIC-TEX affect proteases and more frequently adhesion molecules in v6kd and Tsp8kd cells. CIC-TEX often promote protease inhibitor upregulation. Besides matrix binding molecules, the linkage to the actin cytoskeleton and binding to cadherin is dominating. Altered adhesion molecule-promoted signaling frequently proceeds directly via activated integrins, RTK and GPCR

DS confirmed the engagement of Tsp8 and v6 in adhesion/migration and kd cell deficit correction by CIC-TEX and unraveled an abundance of upregulated cadherin-binding mRNA and of protease inhibitors.

### Attacking CIC-TEX

Taking the strong CIC-TEX impact on Non-CIC tumor progression, CIC-TEX blocking could provide a mean improving adjuvant PaCa therapy. TEX-Tsp8 most efficiently binding targets [28], CIC-TEX were blocked by an anti-Tsp8 antibody (CO029), not captured by xenogeneic host cells. CIC-TEX-promoted signal transduction activation was attacked by GEM, a standard drug in adjuvant PaCa treatment [60].

Nude mice received a sc A818.4-v6kd cell injection and 2-times/wk. CIC-TEX, iv. Where indicated, mice were weekly treated with GEM or CO029. The survival time of CIC-TEX-treated mice was significantly reduced. GEM and CO029 sufficed coping with the impact of CIC-TEX (Fig. 7a). CIC-TEX-promoted tumor cell dissemination in PB, LN and lung was mitigated in GEM-treated mice. CO029 additionally affected settlement in the BM (Fig. 7b).

**Fig. 7:** Binding and RTK inhibition for blocking CIC-TEX activity as adjuvant PaCa therapy. Mice received an ot (A818.4-v6kd) or a sc (A818.4) tumor cell injection and weekly the RTK inhibitor GEM (iv) or anti-Tsp8 (CO029) (iv). **a** Survival time and mean survival time of v6kd-TB mice (intrapancreatic) treated with CIC-TEX (2x/wk) and GEM or CO029 (1x/wk). **b** Recovery of disseminated tumor cells in cultures of dispersed organs at autopsy. **c** Tumor growth rate, survival time and mean survival time of sc A818.4-TB mice, treated with GEM or CO029; **d** disseminated tumor cell recovery in cultures of dispersed organs at autopsy; **a**-**d** p-values for the mean survival time and the numbers of organs containing dispersed tumor cells (after Bonferroni-Holm correction) of GEM- or CO029-treated compared to untreated v6kd-TB and CIC-TEX-treated-TB or wt-TB are indicated. **e**,**g**,**i**,**k**,**l** Flow-cytometry of dispersed tumor cells and BMC of untreated and GEM- or CO029-treated A818.4-TB mice evaluating CIC, angiogenic, apoptosis, proteolysis, adhesion (only tumor cells) marker expression and MDSC (CD11b + Gr1+) (only BMC); mean % stained cells±SD (3 mice), significant differences by GEM- or CO029-treatment: *. **f**,**h**,**j** Immunohistology of A818.4 shock-frozen tumor sections from untreated, GEM- or CO029-treated mice stained for CIC markers, VEGFR2, VEGFR3, CD31, MMP2 and TIMP1 (scale bar: 100 μm). GEM and CO029 weakly affect tumor growth and strongly tumor cell dissemination. Ex vivo analysis indicates that GEM and CO029 act independently. GEM primarily affects tumor cell apoptosis, proteases and MDSC expansion, CO029 treatment is accompanied by a reduction in (Tsp8-associated) CIC markers and compromises (lymph)angiogenesis

To mimic the clinical situation, mice received sc A818.4 cells and weekly GEM or CO029, iv. GEM retarded tumor growth early after application, CO029 became efficient after 4-5wk, GEM and CO029 significantly delaying tumor growth (Fig. 7c). More impressive was the interference with tumor cell dissemination. Settlement in draining LN was prevented in 2, recovery in the PB in 3 of 6 mice. Particularly CO029 potently coped with settlement in BM and lung. Tumor cell dissemination in GEM or CO029-treated mice, evaluated in ex vivo cultures, was significantly reduced (Fig. 7d).

Stem cell marker, angiogenesis-, apoptosis-, proteolysis- and adhesion-related molecule expression was evaluated 6wk after A818.4 application by flow-cytometry and at autopsy by immunohistochemistry. CO029 affected Tsp8 and associated CD104 expression in the primary tumor and the BM (Fig. 7e), reduced expression being also seen at autopsy. An impact of GEM on expression of the CIC-markers v6, Tsp8, CD104 and CD184 in tumor tissue became apparent only by immunohistochemistry performed with shock-frozen tumor tissue at autopsy (Fig. 7f). Only CO029 affected VEGFR3 expression in tumor cells and BMC (Fig. 7g). At autopsy angiogenesis was reduced in tumors of GEM- and CO029-treated mice; CO029 sufficed for mitigating lymphangiogenesis (reduced VEGFR3 expression), which might explain the stronger impact of Tsp8 on metastatic settlement (Fig. 7h). Only GEM application was accompanied by an increase in apoptotic cells (AnnV+ and PI+) and prominently increased TIMP1 expression. Immunohistochemistry at autopsy revealed a slight MMP2 reduction in GEM- and CO029-treated mice that was not seen in flow-cytometry, while TIMP1 upregulation by GEM was confirmed (Fig. 7i,j). Both GEM and CO029 promoted a minor reduction of some integrins and CD56. Tumor cell dissemination-facilitating myeloid-derived suppressor cells (MDSC) were strongly reduced in the BM of GEM-treated mice (Fig. 7k,l).

Briefly, GEM and CO029 counterbalance several CIC-TEX-initiated tumor progression-promoting effects, CO029 most efficiently interfering with tumor cell dissemination, whereas GEM drives apoptosis and affects hematopoiesis. Promising for combining anti-Tsp8 treatment with chemotherapy, the therapeutic effects of GEM and CO029 are independent.

## Discussion

CIC-TEX promote tumor progression affecting host cells and Non-CIC [4, 8, 61], the mode of CIC-TEX modulating targets and an active CIC marker contribution being debated. DS of CIC-TEX, human v6kd and Tsp8kd PaCa Non-CIC and v6kd and Tsp8kd Non-CIC cocultured with CIC-TEX and functional in vitro and in vivo controls enlightened the contribution of v6 and Tsp8 to a range of CIC activities as well as to central aspects of CIC-TEX operation, particularly CIC-TEX content likely promoting a switch in the activation state of central signaling components. The model and our conclusions will be discussed.

### CD44v6kd and Tsp8kd non-CIC and CIC-TEX uptake

CD44v6kd and Tspan8kd PaCa lines can be considered as Non-CIC due to the loss in metastatic capacity [32–34]. This finding on the one hand strengthens v6 and Tsp8 being CIC-biomarkers and on the other hand allowed unraveling their contribution(s) to the metastatic process. Overlapping activities of two apparently independent CIC markers are due to the association in invagination prone TEM, Tsp8 playing a prominent role in TEX biogenesis and targeting and v6 in vesicle loading [26, 28, 33, 62]. Joint loss of activities is endorsed by v6 regulating Tsp8 transcription [32]. Furthermore, CIC-TEX and kd cells originating from one parental clone facilitates coordinating molecular and functional changes, strengthening the suitability of these CIC-marker kd models evaluating CIC-TEX activities of v6 and Tsp8.

CIC-TEX uptake by v6kd and Tsp8kd cells is unimpaired. Uptake in the xenogeneic system by EC and monocytes, to be interpreted with caution, nonetheless reinforces the CIC-TEX - host crosstalk [61, 62]. CIC-GFP supporting at a distant site injected v6kd Non-CIC growth after 4wk and weak GFP expression at autopsy in ~ 10% of v6kd Non-CIC pointed towards released GFP-TEX activity, affirmed by increased recovery of disseminated v6kd and Tsp8kd Non-CIC in CIC-TEX-treated mice. Thus, v6kd and Tsp8kd cells take-up function-relevant CIC-TEX.

### Deep sequencing as a tool elaborating the mode of CIC-TEX activity

CIC-TEX target modulation could be due to the liberated TEX content or, not mutually exclusive, CIC-TEX binding-promoted target cell activation or the TEX content acting as a hub [14, 61]. The latter suggestions are supported by the small Exo plasma hosting limited amounts of proteins, RNA and DNA and by Exo derived from cell clones distinctly affecting different targets [62].

DS was performed with CIC-TEX, untreated and CIC-TEX-treated v6kd and Tsp8kd cells. Due to the coculture components relatedness, CIC-TEX uptake provoked a limited number of coculture-initiated altered mRNA and miRNA recoveries in v6kd and Tsp8kd Non-CIC. DS of Capan1 sphere-derived CIC-TEX, Capan1-v6kd cells and CIC-TEX-treated Capan1-v6kd cells revealed concordant results in > 90% (signal strength cutoff: ≥1000), data not shown for clarity of presentation.

Functional assignment of distinctly recovered mRNA in CIC-TEX-treated v6kd and Tsp8kd cells showed dominant engagement in signaling, transport, transcription and translation. However, neither increased nor decreased mRNA correlated with recovery in CIC-TEX. Thus, changed recovery after coculture does not reflect the TEX content, which also accounts for changed miRNA recovery. Instead, recovery of predicted targets of distinctly recovered cellular miRNA inversely correlated in ≥50%. miRNA-repressed or -released mRNA were mainly engaged in metabolism, signaling and transcription, assignments based on few miRNA-mRNA pairs may not essentially be representative, yet fit to distinctly recovered mRNA in CIC-TEX-treated v6kd and Tsp8kd Non-CIC. One also should take the possibility into account that the activity of TEX miRNA on cellular mRNA translation is missed by the evaluation of mRNA. As after 48 h–72 h coculture the cellular miRNA and the predicted mRNA level inversely correlated in > 50%, we suggest that the coculture period sufficed for covering the impact of miRNA on mRNA translation. Nonetheless, this option should be further explored. Finally, long noncoding (lnc)RNA needs mentioning discussing mRNA release from repression. Abundant lncRNA frequently act as miRNA sponges [63], but current knowledge does not allow a systemic integration into miRNA interfering with mRNA translation.

DS uncovered CIC-TEX more strongly affecting mRNA and miRNA in v6kd than Tsp8kd Non-CIC, which is due to v6 engagement in RTK and transcription factor activation, alternative splicing and miRNA processing [16, 33, 43, 64, 65]. This finding is not opposing a Tsp8kd and a v6kd similarly affecting tumor progression [25, 65, 66], the impact of a Tsp8kd being due to tetraspanin engagement in TEX-biogenesis and -binding/uptake [28, 32, 34].

DS analysis pointing towards CIC-TEX binding-initiated target cell activation and CIC-TEX content transfer acting as a hub was confirmed in vitro and in vivo for selected, tumor progression-associated processes at the protein level.

### CIC-TEX-promoted v6kd and Tsp8kd non-CIC activation, apoptosis-resistance, EMT, motility and tumor progression

Protein analysis of CIC-TEX-treated v6kd and Tsp8kd Non-CIC uncovered RTK upregulation including in v6kd cells Met and EphA4, both interacting with and activated by v6 binding [67, 68]. Occasional cytoplasmic signaling molecule activation after coculture with kd-TEX obviates an exclusive CIC-TEX contribution. Nonetheless, confirming in vitro studies, v6kd tumor ex vivo analysis from CIC-TEX-treated mice additionally uncovered MAPK pathway activation [69], missed after in vitro coculture.

Pathway analysis of upregulated miRNA targets in CIC-TEX-treated v6kd and Tsp8kd Non-CIC backed some miRNA engagement in CIC-TEX-initiated signaling, the main target being Spry4, inhibiting beside others the MAPK pathway [37, 70]. More abundant were upregulated mRNA, correlating with reduced miRNA recovery. Notably, the majority of predicted mRNA being targets of more than one miRNA, like CDK6, DCBLD2, GOLT1B (Golgi transport 1B), GTF2F2 (general transcription factor IIF subunit 2), HES7 (hes family bHLH transcription factor 7), MBP (myelin basic protein), PMAIP1 and PPP3CA, are engaged in cancer-related signaling pathways (reviewed in [71]).

Briefly, CIC-TEX initiate v6kd and Tsp8kd Non-CIC modulation by suppressing or activating signaling pathways and by launching miRNA processing or silencing with concomitant mRNA repression/release of repression. This powerful networking underscores CIC-TEX-promoted modulation of signaling in v6kd and Tsp8kd Non-CIC as hub for regaining CIC-features.

CIC-TEX, hardly affecting components of receptor-mediated apoptosis or the mTOR/Pten pathway, promoted upregulation of ID1 (inhibitor of DNA binding 1, HLH protein), PIM1 and PIM3 (Proto-oncogene, serine/threonine kinase-1, − 3), negative regulators of apoptosis [54, 72–74]. However, DS revealed significant upregulation of 4 drug transporters in CIC-TEX-treated v6kd cells and CIC-TEX-promoted MDR1 expression was miRNA-independent. CD44 plays a central role in ABC regulation [75] and stem cell Exo / CIC-TEX confer drug resistance [76]. At least in the context of v6kd Non-CIC, TEX-promoted ABC upregulation is the dominating mechanism in transferring apoptosis resistance. A weak coculture-induced effect on apoptosis resistance of Tspan8kd cell may rely on PI3K/Akt pathway activation.

There were few possibly miRNA-related changes in apoptosis resistance. We already mentioned that the most prominent targets, like p21, DHCR24, Clu, NGFR, SFN, STAT1, PMAIP1, EMP1, VEGFB and TGM, the only mRNA selectively affected in Tspan8kd cells [55], have multiple functions [44–53], one of the activities of the heat shock protein-similar chaperone Clusterin being apoptosis inhibition by interfering with Bax activation and cytochrome C release [45], BAX expression being slightly reduced in CIC-TEX-treated v6kd cells. Also, EMP1, reported to be downregulated in cancer, can upregulate Casp9 [52]. However, none of these possibly miRNA-regulated mRNA were engaged in receptor promoted apoptosis.

Thus, a major contribution of CIC-TEX to strengthen v6kd apoptosis-resistance relies on ABC transporter upregulation. A minor input by PI3K/Akt pathway components, displaying pronounced phosphorylation, will be missed by DS analyses.

EMT or partial EMT induction is a central feature of CIC [77, 78] and involves CIC-marker expression [79] including CD44 [80]. The confirmation for CD44v6, Tspan8 [4, 31, 32] and CD133 strengthening their definition as CIC-biomarkers. From the classical EMT markers, only N-cadherin [81] was affected by the v6kd and the Tsp8kd, reduced expression becoming corrected in vitro and in vivo by CIC-TEX. Notably, an unexpectedly high number of up- or downregulated mRNA after CIC-TEX coculture is engaged in transcription, translation, Wnt, Nanog or Notch signaling, some of these mRNA being also targets of CIC-TEX coculture-affected miRNA, downregulated miRNA mostly repressing Wnt and NOTCH signaling-engaged mRNA. At the protein level, CIC-TEX induced a partial NOTCH, Nanog and Twist rescue, showing pronounced v6 and Tsp8 colocalization. Flow-cytometry indicated a Slug, Snail, Twist and Wnt5a/b rescue in CIC-TEX-treated v6kd cells. The findings, in line with EMT-related transcription factors assisting tumor progression [78], reinforce the v6 contribution to Wnt, NOTCH and Nanog activation and to miRNA processing [17, 18, 21, 22, 82]. These CIC-TEX activities could rely on the abundant recovery of E2F transcription factor, histone proteins and RISC components in CIC-TEX [83, 84]. Whether the transferred proteins act autonomously or as hub, awaits clarification. All required components being available in Non-CIC and Exo-induced EMT being restricted to embryonic development and tumor cells [85], an initiating CIC-TEX trigger may be dominating.

Controlling by DS the CIC-TEX contribution to migration promoting activity (Fig. 6) [25, 32], two observations, missed at the protein level, need mentioning. A comparably high number of protease inhibitors became upregulated by CIC-TEX treatment. Increased laminin, collagen and FN matrix protein expression in CIC-TEX-treated v6kd and Tsp8kd Non-CIC suggests a feedback loop to guarantee sufficient extracellular matrix (EMC) organization for guiding migrating tumor cells. Furthermore, a high number of mRNA engaged in cadherin-promoted adhesion became upregulated by CIC-TEX treatment. E-cadherin expression, though not consistently observed, is supposed to become reduced during EMT [81]. Occupying E-cadherin by different ligands, preventing homophilic adhesion, could fulfill a similar task as downregulation. Taking into account membrane integrated and actin binding components, DS confirmed the contribution of CIC-TEX in promoting a motile phenotype of v6kd and Tsp8kd Non-CIC, integrins, their ECM ligands and cytoskeleton reorganization being important players.

### Blocking CIC-TEX mitigates the impact on targets

Drug combinations improved adjuvant chemotherapy efficacy in PaCa, success still being unsatisfactory [37]. CIC-TEX contributing to poor PaCa prognosis, we and others explored a CIC-TEX-uptake blockade of the major PaCIC-TEX targeting molecule Tsp8 [28–30]. In view of the impressive activation of RTK by CIC-TEX the kinase inhibitor GEM [60] was used as an alternative option. We confirmed complementation of these two adjuvant therapies. Both GEM and CO029 slightly prolonged the survival time and strongly impaired tumor cell dissemination. Only CO029 affected Tsp8-associated CIC biomarker expression and reduced tumor cell recovery in the BM. GEM predominantly supported apoptosis-susceptibility, protease expression and in the BM a shift towards MDSC. Angiogenesis-related receptor expression was affected by both, lymphangiogenesis receptor expression predominantly in CO029-treated mice.

The supplementing activities of GEM and CO029, antibody application not being burdened by severe side effects, might considerably improve PaCa adjuvant therapy.

## Conclusions

CIC-TEX strongly influence v6kd and Tsp8kd Non-CIC, predominantly affecting signaling, transcription, translation, but also miRNA processing with a feedback on mRNA translation. The v6 CIC marker, engaged in all these processes, takes the lead. Unraveling CIC-TEX binding/transfer likely acting as hub will have profound bearing on understanding the crosstalk between exosomes and targets and be most helpful envisaging outsmarting CIC-TEX, a blockade of CIC-TEX uptake via anti-Tsp8 offering an independent, additive adjuvant therapeutic (Fig. 8).

**Fig. 8:** Summary on the importance of CD44v6 and Tspan8 on CIC-TEX-promoted Non-CIC reprogramming and potential therapeutic interference. CIC-TEX promote a shift towards stem cell features in v6kd and Tsp8kd Non-CIC, CIC-TEX binding/transfer acting as a hub. The v6 importance relies on initiating activation of signal transduction and contributing to mRNA processing. Tspan8 is central in CIC-TEX communication. The complementing v6 and Tsp8 activities open new adjuvant therapeutic options by blocking CIC-TEX binding/uptake and by interfering with CIC-TEX-promoted Non-CIC activation. (CAM: cell adhesion molecules, EMT: epithelial mesenchymal transition, RTK: receptor tyrosine kinases)

## Additional file

Additional file 1: **Table S1.** Alphabetic list of gene symbols. **Table S2.** Antibodies, reagents, primers. **Table S3.** The impact of CIC-TEX on mRNA recovery in CD44v6kd and Tspan8k cells. **Table S4.** The impact of CIC-TEX on miRNA recovery in CD44v6kd and Tspan8k cells. **Table S5.** Correlation between upregulated miRNA and downregulated mRNA. **Figure S1.** TEX characterization and in vivo distribution of CIC-TEX. **Figure S2.** Differences in the mRNA profile of A818.4, −CD44v6kd and -Tspan8kd cells and TEX and the impact of CIC-TEX on CD44v6kd and Tspan8kd cells. **Figure S3.** Distinct miRNA recovery in wt-TEX versus CD44v6kd and Tspan8kd TEX and in kd cells cocultured with CIC-TEX. **Figure S4.** CIC-TEX-initiated changes in RTK and downstream signaling molecules in Tspan8kd cells and mRNA release from repression by reduced miRNA expression in CD44v6kd and/or Tsp8kd cells. **Figure S5.** CIC-TEX-promoted changed miRNA recovery and predicted target mRNA engaged in apoptosis. (PDF 4703 kb)

## Abbreviations

ABC: ATP binding cassette
BM/BMC: Bone marrow/bone marrow cells
CIC: Cancer-initiating cell
Dio/SP-DioC_18_(3): 3,3′-dioctadecyl-5,5′-di(4-sulfophenyl)oxacarbocyanine
DS: Deep sequencing
EC: Endothelial cells
ECL: Enhanced chemiluminescence
ECM: Extracellular matrix
EMT: Epithelial-mesenchymal transition
Exo: Exosomes
FN: Fibronectin
GEM: Gemcitabine
GFP: Green fluorescence protein
IPA: Ingenuity program analysis
iv: Intravenously
kd: Knockdown
LB: Latex beads
LN/LNC: Lymph node/lymph node cells
MDSC: Myeloid-derived suppressor cells
Mϕ: Macrophage
ot: Orthotopic
PaCa: Pancreatic cancer
PB/PBL: Peripheral blood/peripheral blood leukocytes
PEC: Peritoneal exudate cells
PI: Propidium iodine
qRT-PCR: Quantitative real time polymerase chain reaction
RTK: receptor tyrosine kinase
SC: stem cells
sc: subcutaneously
SpC: spleen cells
TB: tumor bearer
TEM: tetraspanin-enriched microdomains
TEX: Tumor exosomes
Tsp8: Tspan8
v6: CD44v6
WB: Western blot
wt: Wild type

## Footnotes

1 For full names of synonyms please see Additional file 1: Table S1, providing an alphabetic list of synonyms
